# Mathematical Analysis of COVID-19 Transmission Dynamics Model in Ghana with Double-Dose Vaccination and Quarantine

**DOI:** 10.1155/2022/7493087

**Published:** 2022-07-28

**Authors:** Philip N. A. Akuka, Baba Seidu, C. S. Bornaa

**Affiliations:** ^1^Department of Mathematics, Bongo Senior High School, Bongo UE/R, Ghana; ^2^Department of Mathematics, School of Mathematical Sciences, C. K. Tedam University of Technology and Applied Sciences, Navrongo, Ghana; ^3^Department of Mathematics and ICT Education, School of Science, Mathematical and Technology Education, C. K. Tedam University of Technology and Applied Sciences, Navrongo, Ghana

## Abstract

The discovery of vaccines for COVID-19 has been helpful in the fight against the spread of the disease. Even with these vaccines, the virus continues to spread in many countries, with some vaccinated persons even reported to have been infected, calling for administration of booster vaccines. The need for continued use of nonpharmaceutical interventions to complement the administration of vaccines cannot therefore be overemphasized. This study presents a novel mathematical model to study the impact of quarantine and double-dose vaccination on the spread of the disease. The local stability analysis of the COVID-19-free and endemic equilibria is examined using the Lyapunov second technique. The equilibria are found to be locally asymptotically stable if *ℛ*_0_ < 1 and *ℛ*_0_ > 1, respectively. Besides other analytical results, numerical simulations are performed to illustrate the analytical results established in the paper.

## 1. Introduction

Coronavirus is an infectious disease caused by a novel strain of virus which originated in Wuhan China, in late March 2019. It was diagnosed in three patients with pneumonia connected to a cluster of acute respiratory illness. As of May 21, 2022, Ghana recorded 161,370 confirmed cases, 159,881 recoveries, and 1,445 deaths [1]. The transmission routes of the virus include environment-to-human and human-to-human. The virus is spread by a close contact (susceptible individual) with an infected person who sneezes, or cough, or by an infected environment such as door holdings, curtains, and cutlery. Some common symptoms of COVID-19 infection include dry cough, fever, fatigue, breathing difficulty, and bilateral lung infiltration in severe cases similar to those caused by SARS-CoV and MERS-CoV infections [2]. Mostly, the infected people develop symptoms within an incubation period ranging from 2 to 14 days [3]. Currently, in Ghana, the combination of azithromycin, vitamin C, zinc, and some fever and pain killer medications seems to be working. Several measures have already been put in place which include travel bans, social distancing, use of facemask, and personal hygiene through frequent hand washing and use of appropriate hand sanitizers [4]. Despite efforts being made to curb the spread of the COVID-19 disease, the disease is still endemic in many parts of the world including Ghana. In early 2020, several companies began to develop vaccines against the COVID-19 virus, and a number of vaccines have been successfully developed. These vaccines have proven to be highly efficacious against COVID-19 (estimated at 91.6%,  95%, 82%,  and 94.1% for Sputnik V, Pfizer, AstraZeneca, and Moderna, respectively) [5–8]. Since a large number of people in the world need to be vaccinated to reduce the spread and mortality, vaccines are in limited supply. Developing countries find it difficult to secure large quantities of vaccines, thereby leading to a small portions of the population being vaccinated. As of May 24, 2022, Ghana Health Service administered a total of 15,032,815 vaccine doses (with 9,724,157 persons receiving at least 1 dose and 6,329,702 persons fully vaccinated) [1]. One needs to take double-dose shots of the vaccine to be fully vaccinated.

A lot of research has been conducted employing mathematical modelling to understand dynamics of the disease and to propose strategies of combatting it [9]. Specifically, [10] used a mathematical model combined with an optimization algorithm to determine optimal allocation strategies with one and two doses of vaccine to minimize five metrics of disease burden under various degrees of viral transmission. They suggested that it is crucial to find out the efficacy and durability of single-dose vaccines, as mixed or single-dose vaccination may have the potential to contain the pandemic much more quickly. [11] studied the nature of the virus, in which they developed and presented a review on the study of finding an effective vaccine for this new coronavirus. A new mathematical model formulated by [12] to study the global dynamics of COVID-19 revealed that, in India and Pakistan, the ratio of transmission and death rate is fast as compared to the other two countries (Bangladesh and Sri Lanka) because huge population produces greater chance to more people infected. [13] formulated and qualitatively analyzed a COVID-19 mathematical model, taking into consideration the available therapeutic measures, vaccination of susceptible, and treatment of hospitalized/infected individuals. The results showed that vaccination and treatment are very effective in mitigating the spread of COVID-19 and concurrently applying personal preventive measures (nonpharmaceutical public health interventions) such as face masks, hand washing, and social distancing should continue to be encouraged. [14] research showed that, when self-quarantined is adopted, then the process may go on reverse direction and infection will be decreasing and hence healthy community may be restored. In [15], the results show that the trend of epidemics mainly depends on quarantined and suspected cases. It will reveal that it is important to continue enhancing the quarantine and isolation strategy and improving the detection rate in mainland China. To the best of our knowledge, none of the literature has considered double-dose vaccination and quarantine. Therefore, this study develops a deterministic compartmental COVID-19 model which incorporates double-dose vaccination and quarantine to simulate the prevalence of COVID-19 disease in Ghana. The rest of the paper is organized as follows. The proposed model is formulated in Section 2, and analytical analysis is presented in Section 3. Numerical simulations performed to support the analytical results are presented in Section 4. The conclusion is presented in Section 5.

## 2. Model Formulation

Annas et al. [16] proposed the following SEIR model to study the impact of isolation and vaccination on the spread of COVID-19 in Indonesia:

(1) $$\begin{array}{c} \left.\begin{array}{c} \frac{\text{d}S}{\text{d}t}=\gamma -\left(\nu +\delta +\beta I\right)S,\\ \frac{\text{d}E}{\text{d}t}=\beta IS-\left(\delta +\mu \right)E,\\ \frac{\text{d}I}{\text{d}t}=\mu E-\left(\alpha +\delta +\delta_{i}\right)I,\\ \frac{\text{d}R}{\text{d}t}=\alpha I+\nu S-\delta R. \end{array}\right\} \end{array}$$

In this paper, the work of Annas et al. [16] is extended to study the impact of quarantine and double-dose vaccination for the COVID-19 transmission in Ghana. The total population (*N*) is divided into the following epidemiological classes: susceptible (individuals who are uninfected but may get infected upon contact with the infectious agent), *S*(*t*) (individuals who have received the first dose of vaccine), *V*_1_(*t*) (individuals who have received the second dose of vaccine), *V*_2_(*t*) (exposed individuals—individuals who are exposed to the virus), *E*(*t*) (individuals who are exposed and have been identified and quarantined), *Q*(*t*) (individuals who are infected and infectious), *I*(*t*) (individuals who have successfully recovered from infection), and *R*(*t*). It has been observed that the rate of infection among those who have been vaccinated is lower than those who have not been vaccinated. The total population size *N*(*t*) is thus given by *N*(*t*) = *S*(*t*) + *V*_1_(*t*) + *V*_2_(*t*) + *E*(*t*) + *Q*(*t*) + *I*(*t*) + *R*(*t*). Recruitments into the population are assumed to be from only susceptibles at rate *γ*. The natural death and COVID-19-induced death rates are given as *δ* and *δ*_*i*_, respectively. Susceptible individuals are assumed to receive first COVID-19 vaccination and move to the vaccinated compartment (*V*_1_) at rate *π*. Single-dose-vaccinated persons lose protection from COVID-19 and rejoin the susceptibles at rate *ε*, while those who receive a second dose move to the *V*_2_ compartment at rate *τ*. The parameter *g* is assumed to be the waning rate of immunity following double vaccination. Susceptible individuals may be infected at rate *βS*(*I* + *E*) following effective contact with viral sources. Those who are exposed are quarantined at a rate *ω*, and it is assumed that a proportion *f* of the quarantined recovers at rate *fκ*, while the remainder join the infected class at a rate (1 − *f*)*κ*. Those who are exposed become infectious at a rate *μ*, and those with clinical symptoms recover at rate *α*. Those who recover may lose immunity at some rate *σ* and move back to the susceptible compartment. The dynamics described so far are presented in Figure 1. The description of the model variables and parameters are presented in Table 1.

The dynamics of COVID-19 described thus far is represented by the following system of nonlinear differential equations:

(2) $$\begin{array}{c} \left.\begin{array}{c} \frac{\text{d}S}{\text{d}t}=\gamma +\varepsilon \left(V_{1}+\left(1-g\right)V_{2}\right)+\sigma R-\beta \left(I+E\right)S-\left(\pi +\delta \right)S,\\ \frac{\text{d}V_{1}}{\text{d}t}=\pi S-\beta \left(I+E\right)\left(1-\eta_{1}\right)V_{1}-\left(\varepsilon +\delta +\tau \right)V_{1},\\ \frac{\text{d}V_{2}}{\text{d}t}=\tau V_{1}-\beta \left(I+E\right)\left(1-\eta_{2}\right)V_{2}-\left(\delta +\left(1-g\right)\varepsilon \right)V_{2},\\ \frac{\text{d}E}{\text{d}t}=\beta \left(I+E\right)\left[S+\left(1-\eta_{1}\right)V_{1}+\left(1-\eta_{2}\right)V_{2}\right]-\left(\omega +\delta +\mu \right)E,\\ \frac{\text{d}Q}{\text{d}t}=\omega E-\left(\delta +\kappa \right)Q,\\ \frac{\text{d}I}{\text{d}t}=\mu E+\kappa \left(1-f\right)Q-\left(\alpha +\delta +\delta_{i}\right)I,\\ \frac{\text{d}R}{\text{d}t}=\alpha I+f\kappa Q-\left(\sigma +\delta \right)R,\\ \text{with nonnegative initial conditions}. \end{array}\right\} \end{array}$$

In the subsequent discussions, where necessary, the following conventions are used:

(3) $$\begin{array}{c} \begin{array}{c} k_{1}=\left(\pi +\delta \right),\\ k_{2}=\left(\varepsilon +\delta +\tau \right),\\ k_{3}=\left(\delta +\left(1-g\right)\varepsilon \right),\\ k_{4}=\left(\omega +\delta +\mu \right),\\ k_{5}=\left(\delta +\kappa \right),\\ k_{6}=\left(\alpha +\delta +\delta_{i}\right),\\ k_{7}=\left(\sigma +\delta \right),\\ \Gamma =k_{2}k_{3}k_{1}-\pi \varepsilon \left(\left(1-g\right)\tau +k_{3}\right). \end{array} \end{array}$$

## 3. Qualitative Properties

### 3.1. Positivity and Boundedness of Solutions of Model (2)

**Lemma 1 .**

The following result concerns the nature of solutions of model (2).

1. If the initial values of state variables of model (2) are nonnegative, then all future values of state variables are also positive
2. The set defined by *Ω* ⊂ ℝ_+_^7^ defined by *Ω* = {(*S*, *V*_1_, *V*_2_, *E*, *Q*, *I*, *R*) ∈ ℝ_+_^7^|0 ≤ *N*(*t*) ≤ (*γ*/*δ*)} is a positively invariant region for model (2)

**Proof**

It should be noted that the right-hand side of all components of model (2) is continuous and also locally Lipschitz at *t* = 0. Therefore, every nonnegative initial conditions of model (2) has a unique nonnegative solution in ℝ_+_^7^ for all *t* > 0, concluding the first part of the lemma.

Furthermore, it is easy to show that if *X* = (*S*(*t*),  *V*_1_(*t*),  *V*_2_(*t*), *E*(*t*), *Q*(*t*), *I*(*t*), *R*(*t*)) ∈ ℝ_+_^7^ and *X*_*i*_ = 0, then (d*X*_*i*_/d*t*) ≥ 0. Therefore, from Theorem A.4 of [17], the region ℝ_+_^7^ is positively invariant under the flow induced by model (2).

Now, summing all equations in model (2) gives

(4) $$\begin{array}{c} \frac{\text{d}N}{\text{d}t}=\gamma -\delta \;N-\delta_{i}I\leq \gamma -\delta \;N, \end{array}$$

so that we have $\lim\underset{t⟶\infty }{\sup}N\left(t\right)\leq \left(\gamma /\delta \right)$. Since *N*(*t*) is bounded, then each component of *X* is also bounded, and hence, the feasible set of the model is given by *Ω*.

As for the invariance of *Ω*, it can be noted that from (d*N*/d*t*) ≤ *γ* − *δ* *N*, it is easy to show that (d*N*/d*t*) < 0 whenever *N* > (*γ*/*δ*). This shows that *Ω* is positively invariant under the flow induced by model (2), concluding the proof of the second part of the lemma.

Therefore, model (2) is mathematically and epidemiologically well posed [18] in *Ω*, and all analyses are therefore considered to be inside of *Ω*.

### 3.2. Equilibrium Points of the Model

It is easy to see that model (2) has a COVID-19-free equilibrium point *ε*_0_ = (*S*^0^, *V*_1_^0^, *V*_2_^0^,0,0,0,0), where *S*^0^ = *γ* *k*_2_*k*_3_/Γ, *V*_1_^0^ = *π* *γ* *k*_3_/Γ, and *V*_2_^0^ = *τ* *π* *γ*/Γ.

The basic reproduction number (*ℛ*_0_) is defined as the average number of secondary COVID-19 infections caused by a single COVID-19 case throughout his/her entire period of infectiousness. This threshold is determined using the next-generation matrix technique which defines *ℱ* as transmission matrix and *𝒱* as the transition matrix [19]. The matrices *ℱ* and *𝒱* are given as

(5) $$\begin{array}{c} \begin{array}{c} F=\left(\begin{array}{ccc} B_{0} & 0 & B_{0}\\ 0 & 0 & 0\\ 0 & 0 & 0 \end{array}\right),\\ V=\left(\begin{array}{ccc} k_{4} & 0 & 0\\ -\omega & k_{5} & 0\\ -\mu & -\kappa \left(1-f\right) & k_{6} \end{array}\right), \end{array} \end{array}$$

where *ℬ*_0_ = *β*[*S*^0^ + (1 − *η*_1_)*V*_1_^0^ + (1 − *η*_2_)*V*_2_^0^].

Therefore,

(6) $$\begin{array}{c} {FV}^{-1}=B_{0}\left(\begin{array}{ccc} \frac{1}{k_{4}}+\frac{\mu \;k_{5}+\kappa \;\omega \left(1-f\right)}{k_{5}\;k_{6}\;k_{4}} & \frac{\kappa \;\left(1-f\right)}{k_{5}\;k_{6}} & \frac{1}{k_{6}}\\ 0 & 0 & 0\\ 0 & 0 & 0 \end{array}\right), \end{array}$$

and the basic reproduction number is obtained as the largest eigenvalue of *ℱ𝒱*^−^ and is given by

(7) $$\begin{array}{c} R_{0}=\frac{B_{0}}{k_{4}}\left(1+\frac{\mu \;k_{5}+\kappa \;\omega \left(1-f\right)}{k_{5}k_{6}}\right). \end{array}$$

Let *ε*^∗^ = (*S*^∗^, *V*_1_^∗^, *V*_2_^∗^, *E*^∗^, *Q*^∗^, *I*^∗^, *R*^∗^) be a fixed point of model (2).

Then,

(8) $$\begin{array}{c} \left.\begin{array}{c} S^{*}=\frac{\gamma \;k_{4}\psi_{1}\psi_{2}}{\psi_{1}\psi_{2}\left(k_{1}k_{4}+\left(k_{4}-\psi_{0}\right)\lambda^{*}\right)-\pi \left[\left[k_{4}\varepsilon +\left(1-\eta_{1}\right)\psi_{0}\lambda^{*}\right]\psi_{2}+\tau \left[k_{4}\varepsilon \left(1-g\right)+\left(1-\eta_{2}\right)\psi_{0}\lambda^{*}\right]\right]},\\ V_{1}^{*}=\frac{\pi \;S^{*}}{\psi_{1}},\\ V_{2}^{*}=\frac{\pi \tau S^{*}}{\psi_{1}\psi_{2}},\\ E^{*}=\frac{\lambda^{*}}{k_{4}}\left(1+\frac{\pi \left(1-\eta_{1}\right)}{\psi_{1}}+\frac{\pi \tau \left(1-\eta_{2}\right)}{\psi_{1}\psi_{2}}\right)S^{*},\\ Q^{*}=\frac{\omega }{k_{5}}E^{*},\\ I^{*}=\frac{k_{4}}{B_{0}}\left(R_{0}-\frac{B_{0}}{k_{4}}\right)E^{*},\\ R^{*}=\frac{1}{k_{7}}\left[\frac{\alpha \;k_{4}}{B_{0}}\left(R_{0}-\frac{B_{0}}{k_{4}}\right)+\frac{f\kappa \omega }{k_{5}}\right]E^{*}, \end{array}\right\} \end{array}$$

where

(9) $$\begin{array}{c} \begin{array}{c} \psi_{0}=\sigma \left(\frac{\alpha \;k_{4}}{k_{7}B_{0}}\left(R_{0}-\frac{B_{0}}{k_{4}}\right)+\frac{f\kappa \omega }{k_{5}k_{7}}\right),\\ \psi_{1}=\left(1-\eta_{1}\right)\lambda^{*}+k_{2},\\ \psi_{2}=\left(1-\eta_{2}\right)\lambda^{*}+k_{3}, \end{array} \end{array}$$

and *λ*^∗^ satisfies the following polynomial equation:

(10) $$\begin{array}{c} \left(\Psi_{3}{\left(\lambda^{*}\right)}^{3}+\Psi_{2}{\left(\lambda^{*}\right)}^{2}+\Psi_{1}\lambda^{*}+\Psi_{0}\right)\lambda^{*}=0, \end{array}$$

where

(11) $$\begin{array}{c} \Psi_{3}=\left(1-\eta_{1}\right)\left(1-\eta_{2}\right)\left(\psi_{0}-k_{4}\right),\\ \Psi_{2}=\left(1-\eta_{1}\right)\left(1-\eta_{2}\right)\left(\frac{\beta \;k_{4}\gamma R_{0}}{B_{0}}+{\pi \psi }_{0}-k_{1}k_{4}\right)-\left(k_{4}-\psi_{0}\right)\left[k_{3}\left(1-\eta_{1}\right)+k_{2}\left(1-\eta_{2}\right)\right],\\ \Psi_{1}=\left(\frac{\beta \gamma \;k_{4}R_{0}}{B_{0}}-k_{1}k_{4}\right)\left[k_{3}\left(1-\eta_{1}\right)+k_{2}\left(1-\eta_{2}\right)\right]-k_{2}k_{3}k_{4}+k_{2}k_{3}\psi_{0}+k_{4}\pi \varepsilon \left(1-\eta_{2}\right)+\pi \left(1-\eta_{1}\right)\left(1-\eta_{2}\right)\frac{\beta \gamma \;k_{4}R_{0}}{B_{0}}+{\pi \psi }_{0}\left(k_{3}\left(1-\eta_{1}\right)+\tau \left(1-\eta_{2}\right)\right),\\ \Psi_{0}=k_{4}\pi \varepsilon \left(k_{3}+\tau \left(1-g\right)\right)-k_{1}k_{2}k_{3}k_{4}+\frac{\beta \gamma \;k_{4}R_{0}}{B_{0}}\left(k_{2}k_{3}+k_{3}\pi \left(1-\eta_{1}\right)+\pi \tau \left(1-\eta_{2}\right)\right). \end{array}$$

Equation (10) has four roots, namely, *λ*^∗^ = 0 which corresponds with the disease-free equilibrium and the positive real zeros of the following equation:

(12) $$\begin{array}{c} \Psi_{3}{\left(\lambda^{*}\right)}^{3}+\Psi_{2}{\left(\lambda^{*}\right)}^{2}+\Psi_{1}\lambda^{*}+\Psi_{0}, \end{array}$$

which correspond to the endemic equilibrium of model (2).

Since all parameter values of the model are positive, Ψ_3_ > 0 for *ℛ*_0_ > 1, which implies the existence of at least one positive root for Equation (10). Therefore, the number of positive roots of Equation (10) and the number of endemic equilibrium points of model (2) depend on the signs of Ψ_2_, Ψ_1_, and Ψ_0_.

The following result about the endemic equilibrium of model (2) is thus in the following order.

**Theorem 1 .**

1. There is a critical threshold *ℛ*^∗^ = *ℬ*_0_/*k*_4_ such that model (2) has an endemic equilibrium only when *ℛ*_0_ > *ℛ*^∗^
2. Model (2) has three endemic equilibria whenever Ψ_*i*_ > 0, ∀*i* = 0, 1, 2, 3
3. Model (2) has a unique endemic equilibrium for cases 1, 3, and 4 as given in Table 2

### 3.3. Local Stability of Equilibria

In this section, we investigate the local asymptotic stability of the equilibria.

**Theorem 2 .**

The COVID-19-free fixed point *ε*_0_ of model (2) is locally asymptotically stable whenever *ℛ*_0_ ≤ 1 and unstable otherwise.

**Proof**

The Jacobian matrix of (2) at the COVID-19-free equilibrium point is given by

(13) $$\begin{array}{c} J\left(\varepsilon_{0}\right)=\left[\begin{array}{ccccccc} -k_{1} & \varepsilon & \left(1-g\right)\varepsilon & -\beta \;S^{0} & f\kappa & -\beta \;S^{0} & \sigma \\ \pi & -k_{2} & 0 & -\beta \;\left(1-\eta_{1}\right)V_{1}^{0} & 0 & -\beta \;\left(1-\eta_{1}\right)V_{1}^{0} & 0\\ 0 & \tau & -k_{3} & -\beta \;\left(1-\eta_{2}\right)V_{2}^{0} & 0 & -\beta \;\left(1-\eta_{2}\right)V_{2}^{0} & 0\\ 0 & 0 & 0 & B_{0}-k_{4} & 0 & B_{0} & 0\\ 0 & 0 & 0 & \omega & -k_{5} & 0 & 0\\ 0 & 0 & 0 & \mu & \kappa \;\left(1-f\right) & -k_{6} & 0\\ 0 & 0 & 0 & 0 & f\kappa & \alpha & -k_{7} \end{array}\right]. \end{array}$$

The following is the characteristic polynomial of the Jacobian matrix.

(14) $$\begin{array}{c} \left(\zeta +k_{7}\right)\left(\zeta^{3}+a_{1}\zeta^{2}+a_{2}\zeta +a_{3}\right)\left(\zeta^{3}+b_{1}\zeta^{2}+b_{2}\zeta +b_{3}\right)=0, \end{array}$$

where

(15) $$\begin{array}{c} \begin{array}{c} a_{1}=\frac{\left(\omega \;\kappa \;\left(1-f\right)+\mu \;k_{5}\right)k_{4}+\left(1-R_{0}\right)k_{4}k_{5}k_{6}}{k_{6}k_{5}+\omega \;\kappa \;\left(1-f\right)+\mu \;k_{5}}+k_{5}+k_{6},\\ a_{2}=\frac{\left(k_{6}+k_{5}\right)k_{4}\omega \;\kappa \;\left(1-f\right)+{k_{4}}^{2}\mu \;{k_{5}}^{2}k_{5}\left(1-R_{0}\right)k_{6}\left(\mu +k_{6}+k_{5}\right)}{k_{6}k_{5}+\omega \;\kappa \;\left(1-f\right)+\mu \;k_{5}}+k_{6}k_{5},\\ a_{3}=\left(1-R_{0}\right)k_{4}k_{5}k_{6},\\ b_{1}=k_{1}+k_{2}+k_{3},\\ b_{2}=k_{3}k_{1}-\varepsilon \pi +k_{3}k_{2}+k_{2}k_{1},\\ b_{3}=k_{3}k_{2}k_{1}-\pi \;\varepsilon \left(\tau \left(1-g\right)+k_{3}\right). \end{array} \end{array}$$

It is easy to see that that *b*_2_ > 0 and *b*_3_ > 0, so that all coefficients of the polynomial (14) are positive whenever *ℛ*_0_ ≤ 1. By the Descartes rule of signs, all roots of polynomial (14) are negative. Therefore, *ε*_0_ is locally asymptotically stable whenever *ℛ*_0_ ≤ 1; otherwise, it is unstable, concluding the proof.

### 3.4. Sensitivity Analysis of *ℛ*_0_

Estimates for some parameters are varied one at a time to investigate the impact on the basic reproduction number (*ℛ*_0_). This is done using the normalized forward sensitivity index (NFSI) defined as follows.

The normalized forward sensitivity index of *ℛ*_0_ with respect to the parameter *y* is defined as [22]

(16) $$\begin{array}{c} P_{y}^{R_{0}}=\frac{\partial R_{0}}{\partial y}\times \frac{y}{R_{0}}. \end{array}$$

Using the parameter values in Table 1, the sensitivity indexes of the model parameters determining *ℛ*_0_ are presented in Table 3. The simulation and analysis made are based on data obtained from literature as displayed in Table 1.

In Table 3, the results show that the parameters *β*,  *γ*,  *μ*,  *κ*,  and *ε* have a positive correlation with *ℛ*_0_, which indicates that increasing (decreasing) these parameters will increase the prevalence of COVID-19 disease. On the other hand, the parameters *α*,  *π*,  *τ*,  *ω*,  and *δ*_*i*_ have a negative correlation with *ℛ*_0_, which indicates that increasing (decreasing) these parameters will decrease the prevalence of COVID-19 disease.

### 3.5. Bifurcation Analysis

Let **v** = [*v*_1_ *v*_2_ *v*_3_ *v*_4_ *v*_5_ *v*_6_ *v*_7_] and $w={\left[\begin{array}{ccccccc} w_{1} & w_{2} & w_{3} & w_{4} & w_{5} & w_{6} & w_{7} \end{array}\right]}^{T}$ be the left and right eigenvectors, respectively, of the Jacobian matrix *𝒥*(*ε*_0_). Then,

(17) $$\begin{array}{c} \left.\begin{array}{r} -k_{1}w_{1}+\varepsilon \;w_{2}+\varepsilon \left(1-g\right)w_{3}-\beta \;S^{0}\left(w_{4}+w_{6}\right)+f\kappa \;w_{5}+\sigma \;w_{7}=0,\\ \pi w_{1}-k_{2}w_{2}-\beta \;\left(1-\eta_{1}\right)V_{1}^{0}\left(w_{4}+w_{6}\right)=0,\\ \tau \;w_{2}-k_{3}w_{3}-\beta \;\left(1-\eta_{2}\right)V_{2}^{0}\left(w_{4}+w_{6}\right)=0,\\ -k_{4}w_{4}+B_{0}\left(w_{4}+w_{6}\right)=0,\\ \omega \;w_{4}-k_{5}w_{5}=0,\\ \mu \;w_{4}+\kappa \left(1-f\right)w_{5}-k_{6}w_{6}=0,\\ f\kappa \;w_{5}+\alpha \;w_{6}-k_{7}w_{7}=0. \end{array}\right\} \end{array}$$

From the last three equations in (17), we get

(18) $$\begin{array}{c} \begin{array}{c} \begin{array}{c} w_{5}=\frac{\omega }{k_{5}}w_{4},\\ w_{6}=\left(\frac{\mu \;k_{5}+\omega \kappa \left(1-f\right)}{k_{5}k_{6}}\right)w_{4},\\ w_{7}=\left(\frac{\omega \;f\kappa }{k_{5}k_{7}}+\frac{\alpha \left(\mu \;k_{5}+\omega \kappa \left(1-f\right)\right)}{k_{5}k_{6}k_{7}}\right)w_{4}. \end{array} \end{array} \end{array}$$

Substituting *w*_5_, *w*_6_, and *w*_7_ into the first three equations of (17) gives the following set of equations:

(19) $$\begin{array}{c} \left.\begin{array}{r} -k_{1}w_{1}+\varepsilon \;w_{2}+\varepsilon \left(1-g\right)w_{3}=K_{1}w_{4},\\ \pi w_{1}-k_{2}w_{2}=K_{2}w_{4},\\ \tau \;w_{2}-k_{3}w_{3}=K_{3}w_{4}, \end{array}\right\} \end{array}$$

where

(20) $$\begin{array}{c} \begin{array}{c} K_{1}=\left[\beta \;S^{0}\left(\frac{k_{5}k_{6}+\mu \;k_{5}+\omega \kappa \left(1-f\right)}{k_{5}k_{6}}\right)-\frac{f\kappa \omega }{k_{5}}-\frac{\omega \sigma \;f\kappa }{k_{5}k_{7}}+\frac{\alpha \sigma \left(\mu \;k_{5}+\omega \kappa \left(1-f\right)\right)}{k_{5}k_{6}k_{7}}\right],\\ K_{2}=\beta \;\left(1-\eta_{1}\right)V_{1}^{0}\left(\frac{k_{5}k_{6}+\mu \;k_{5}+\omega \kappa \left(1-f\right)}{k_{5}k_{6}}\right),\\ K_{3}=\beta \;\left(1-\eta_{2}\right)V_{2}^{0}\left(\frac{k_{5}k_{6}+\mu \;k_{5}+\omega \kappa \left(1-f\right)}{k_{5}k_{6}}\right). \end{array}\\ \left.\begin{array}{r} \left[\frac{\varepsilon \;k_{3}}{\tau }+\varepsilon \left(1-g\right)-\frac{k_{1}k_{2}k_{3}}{\pi \tau }\right]w_{3}=\left(K_{1}+\frac{k_{1}k_{2}K_{3}+\tau \;k_{1}K_{2}}{\pi \tau }-\frac{\varepsilon \;K_{3}}{\tau }\right)w_{4},\\ w_{1}=\left(\frac{k_{2}k_{3}}{\pi \tau }w_{3}+\frac{k_{2}K_{3}+\tau \;K_{2}}{\pi \tau }w_{4}\right),\\ w_{2}=\left(\frac{k_{3}}{\tau }w_{3}+\frac{K_{3}}{\tau }w_{4}\right). \end{array}\right\} \end{array}$$

The left eigenvectors of *𝒥*(*ε*_0_) satisfy the following set of equations:

(21) $$\begin{array}{c} \left.\begin{array}{r} -k_{1}v_{1}+\pi \;v_{2}=0,\\ \varepsilon \;v_{1}-k_{2}v_{2}+\tau \;v_{3}=0,\\ \varepsilon \left(1-g\right)v_{1}-k_{3}v_{3}=0,\\ -\beta \left[S^{0}v_{1}+\left(1-\eta_{1}\right)V_{1}^{0}v_{2}+\left(1-\eta_{2}\right)V_{2}^{0}v_{3}\right]+\left(B_{0}-k_{4}\right)v_{4}+\omega \;v_{5}+\mu \;v_{6}=0,\\ f\kappa \;v_{1}-k_{5}v_{5}+\kappa \left(1-f\right)v_{6}+f\kappa \;v_{7}=0,\\ -\beta \;S^{0}v_{1}-\beta \left(1-\eta_{1}\right)V_{1}^{0}v_{2}-\beta \left(1-\eta_{2}\right)V_{2}^{0}v_{3}+B_{0}v_{4}-k_{6}v_{6}+\alpha \;v_{7}=0,\\ \sigma \;v_{1}-k_{7}v_{7}=0. \end{array}\right\} \end{array}$$

From (21), we get

(22) $$\begin{array}{c} \begin{array}{c} v_{1}=0,\\ v_{2}=0,\\ v_{3}=0,\\ v_{7}=0,\\ v_{6}=\frac{B_{0}}{k_{6}}v_{4},\\ v_{5}=\frac{B_{0}\kappa \left(1-f\right)}{k_{5}k_{6}}v_{4}, \end{array} \end{array}$$

where *w*_4_ and *v*_4_ are chosen such that **w**•**v** = 1.

Thus,

(23) $$\begin{array}{c} \left(1+B_{0}\left(\frac{\omega \kappa \left(1-f\right)}{k_{5}^{2}k_{6}}+\frac{\mu \;k_{5}+\omega \kappa \left(1-f\right)}{k_{5}k_{6}^{2}}\right)\right)v_{4}w_{4}=1. \end{array}$$

The bifurcation coefficients are thus obtained as

(24) $$\begin{array}{c} \begin{array}{c} a=\overset{n}{\underset{i,\;j,\;k=1}{\sum }}v_{k}w_{i}w_{j}\frac{\partial^{2}f_{k}}{\partial \;x_{i}\partial \;x_{j}},\\ b=\overset{n}{\underset{i,\;k=1}{\sum }}v_{k}w_{i}\frac{\partial^{2}f_{k}}{\partial \;x_{i}\partial \beta^{*}}, \end{array}\\ a=v_{4}\overset{7}{\underset{i,\;j=1}{\sum }}w_{i}w_{j}\frac{\partial^{2}f_{4}}{\partial \;x_{i}\partial \;x_{j}},\\ f_{4}=\beta \left(x_{4}+x_{6}\right)\left[x_{1}+\left(1-\eta_{1}\right)x_{2}+\left(1-\eta_{2}\right)x_{3}\right]-\left(\omega +\delta +\mu \right)x_{4}. \end{array}$$

The nonzero derivatives in **a** are

(25) $$\begin{array}{c} \frac{\partial^{2}f_{4}}{\partial \;x_{1}\partial \;x_{4}}=\frac{\partial^{2}f_{4}}{\partial \;x_{1}\partial \;x_{6}}=\beta ,\\ \frac{\partial^{2}f_{4}}{\partial \;x_{2}\partial \;x_{4}}=\frac{\partial^{2}f_{4}}{\partial \;x_{2}\partial \;x_{6}}=\beta \left(1-\eta_{1}\right),\\ \frac{\partial^{2}f_{4}}{\partial \;x_{3}\partial \;x_{4}}=\frac{\partial^{2}f_{4}}{\partial \;x_{3}\partial \;x_{6}}=\beta \left(1-\eta_{2}\right),\\ a=2\beta \;\left(w_{6}+w_{4}\right)\left[w_{1}+\left(1-\eta_{1}\right)w_{2}+\left(1-\eta_{2}\right)w_{3}\right]v_{4}. \end{array}$$

Since *v*_1_ = *v*_2_ = *v*_3_ = *v*_7_ = 0 and *f*_5_ and *f*_6_ do not have nonlinear terms, then **b** can be reduced to

(26) $$\begin{array}{c} b=v_{4}\overset{n}{\underset{i=1}{\sum }}w_{i}\frac{\partial^{2}f_{4}}{\partial \;x_{i}\partial \beta^{*}}. \end{array}$$

Also, the nonzero derivatives in **b** are

(27) $$\begin{array}{c} \frac{\partial^{2}f_{4}}{\partial \;x_{4}\partial \beta }=\frac{\partial^{2}f_{4}}{\partial \;x_{6}\partial \beta }=B_{0}. \end{array}$$

Therefore,

(28) $$\begin{array}{c} b=v_{4}\left(w_{6}+w_{4}\right)B_{0}>0. \end{array}$$

Therefore, the nature of the bifurcation depends on the sign of **a**. When *a* > 0, the bifurcation is subcritical (backward), and when *a* < 0, there is forward bifurcation.

## 4. Numerical Simulation and Discussion

In this section, numerical simulations are carried out to support the analytical results and to assess the impact of some model parameters. Numerical simulation for the model of Equation (2) is done using MATLAB R2007b ODE45. The parameter values are given in Table 2, and the initial conditions *S*(0) = 0.98, *V*_1_(0) = 0.02, *V*_2_(0) = 0.01, *E*(0) = 0.2, *Q*(0) = 0, *I*(0) = 0, and *R*(0) = 0.01. The trend of *β* and *μ* on infected population and *π*, *ω*, and *τ* on infected population are given in Figures 2 and 3.

In Figure 4, it is observed that *β*,  *γ*,  and *ε* are positively correlated with *ℛ*_0_, thus increasing (decreasing) *β*,  *γ*,  or *ε* by say 5% will lead to an increase (decrease) in *ℛ*_0_. Similarly, when we increase (decrease) *τ*,  *π*,  *α*,  or *δ*_*i*_ by say 5%, *ℛ*_0_ will decrease (increase). This implies that *τ*,  *π*,  *α*,  and *δ*_*i*_ are negatively correlated with *ℛ*_0_.

Figure 2 shows that the effect of transmission rate (*β*) and progression rate (*μ*) on COVID-19 prevalence. It can be seen in these figures that as the transmission (*β*) and progression rates (*μ*) increase, then COVID-19 prevalence (infected population) increases, which means that those are directly related with COVID-19 outbreak. Efforts needs to be made to reduce the transmission rate (*β*) which can be done through mass vaccination.

Figure 3 shows that the increase in first dose vaccination (*π*), quarantined (*ω*), and second dose vaccination rates (*τ*) decrease the COVID-19 prevalence (infected population) and decrease the risk of an outbreak, which means that these measures should be put in place to minimize the spread of the virus.

## 5. Conclusions

In this paper, a deterministic model is formulated to investigate the spread of COVID-19 in Ghana, taking into account double-dose vaccination and quarantine. Qualitative analysis, bifurcation analysis, and some numerical simulations are conducted on the model. The local stability analysis of the COVID-19-free and endemic equilibria are examined using the Lyapunov second technique. The equilibria are found to be locally asymptotically stable if *ℛ*_0_ < 1 and *ℛ*_0_ > 1, respectively. Figure 3 shows that the disease is expected to become extinct when the basic reproduction number is sufficiently low, which can be achieved by decreasing the parameter *β* or increasing the parameter *τ*. The authors in [16] research showed that isolation and vaccination can reduce the spread of the disease. Sensitivity analysis and numerical simulations confirm that the implementation of double-dose vaccination and quarantine will help minimize the spread of COVID-19. This really implies that, when precautionary measures are put in place, the spread of the virus will be minimized as stated by [23]. Therefore, more education should be done for people to avail themselves for vaccination, and mass vaccination should be done to cover most of the population to reduce spread of COVID-19 in Ghana.

## Figures and Tables

**Figure 1:** Flowchart for COVID-19 model with double-dose vaccination and quarantine.

**Figure 2:** Solution curves depicting the impact of *β* and *μ* on infected population of the COVID-19 model.

**Figure 3:** Solution curves depicting the impact of *π*, *ω*, and *τ* on infected population of the COVID-19 model.

**Figure 4:** Correlation between the reproduction number (*ℛ*_0_) and the model parameters *β*,  *α*,  *ε*,  *π*,  *γ*,  *τ*,  and *δ*_*i*_.

**Table 1:** Parameters estimates of the model.

Para.	Description	Value (per day)	Source
*κ*	Rate at which individuals leave the quarantined class	0.1	[20]
*μ*	Rate of exposed person to infectious	0.3739	Estimated
*α*	Rate of recovery	0.610	Estimated
*β*	Transmission rate	0.0369	Estimated
*δ*	Natural death rate	0.0078	[21]
*δ*_*i*_	COVID-19-induced death rate	0.0045	[1]
*σ*	Immunity loss rate	0.0167	Estimated
*ω*	Rate at which exposed persons are quarantined	0.173	Estimated
*π*	First dose of vaccine rate	0.12	Estimated
*γ*	Recruitment rate	0.23	Estimated
*τ*	Second dose of vaccine rate	0.34	Estimated
*ε*	Rate of waning of immunity after first does	0.6	Estimated
*η*_1_	Efficacy of first dose of vaccine	0.82	[7]
*η*_2_ ≥ *η*_1_	Efficacy of second dose of vaccine	0.82	[7]

**Table 2:** Number of possible positive roots of endemic polynomial in (10).

Case	Ψ_0_	Ψ_1_	Ψ_2_	Ψ_3_	No. of +ve roots of (10)
1	—	+	+	+	1
2	—	+	—	+	0,3
3	—	—	+	+	1
4	—	—	—	+	1
5	+	—	+	+	1,2
6	+	—	—	+	1,2
7	+	+	—	+	1,2

**Table 3:** Sensitivity signs of *ℛ*_0_ to the parameters in Equation (7).

Parameter	Sensitivity index
*β*	+1.000
*γ*	+1.000
*ε*	+0.716
*μ*	+0.324
*κ*	+0.213
*α*	-0.980
*π*	-0.450
*τ*	-0.176
*ω*	-0.123
*δ*_*i*_	-0.007

## Data Availability

The parameter values (data) used to support the findings of this study have been described in subsection 3.4.1.
